The article "Recombinant LH supplementation during IVF cycles with a GnRH-antagonist in estimated poor responders: A cross-matched pilot investigation of the optimal daily dose and timing" was published in 2015. Journal: Mol Med Rep.

# Recombinant LH supplementation during IVF cycles with a GnRH-antagonist in estimated poor responders: A cross-matched pilot investigation of the optimal daily dose and timing

**DOI:** 10.3892/mmr.2015.3904

**Published:** 2015-06-09

**Authors:** SALVATORE GIZZO, ALESSANDRA ANDRISANI, MARCO NOVENTA, SERENA MANFÈ, ALESSANDRA OLIVA, MICHELE GANGEMI, GIOVANNI BATTISTA NARDELLI, GUIDO AMBROSINI

**Affiliations:** Department of Women's and Children's Health, Assisted Reproductive Unit of the Gynecological and Obstetrics Clinic, University of Padua, I-35128 Padua, Italy

**Keywords:** recombinant luteinizing hormone supplementation, poor responders, oocyte quality, embryo quality, pregnancy rate, timing, daily dose

## Abstract

Although it is widely accepted that patients, who are considered poor responders to *in vitro* fertilization (IVF) benefit from recombinant luteinizing hormone (rLH) supplementation during an *in vitro* fertilization cycle, particularly when gonadotropin-releasing hormone (GnRH) antagonist (ant) treatment is used the optimal administration timing and daily dose of rLH remains to be elucidated. The aim of the present study was to investigate the optimal timing of rLH-supplementation to improve ovarian response, embryo quality, endometrial thickness and pregnancy rate in infertile, estimated poor responders to IVF, undergoing GnRH-ant treatment. In addition, the present study aimed to evaluate the optimal daily dose to achieve the same outcomes. A prospective-randomized-cross-matched investigation was performed on 40 patients undergoing a GnRH-ant-treatment-cycle The patients were randomly assigned to either group A (rLH-75 IU/day) or group B (rLH-150 IU/day) and further randomized into subgroup A1/B1, in which rLH was administered at recombinant follicle stimulating hormone (rFSH) administration, and subgroup A2/B2, in which rLH was administered at GnRH-ant administration. Patients who did not become pregnant during the first cycle (35 patients), were treated a second time, cross-matched for groups and subgroups. Improved ovarian response, embryo quality and pregnancy rate were achieved by administering rLH at 150 IU/day, starting from GnRH-ant administration, independently from the total rLH dose administered. Improved endometrial thickness at oocyte retrieval day was achieved by administering rLH at 150 IU from the start of rFSH administration. These data led to the hypothesis that ovarian responses are affected by the timing of administration more than the total-dose of rLH. The optimal window to administer rLH appears to be the mid-to-late follicular phase, despite the fact that rLH-supplementation in the early follicular phase appeared to increase endometrial thickness and to enhance its morphology. Standardization of the optimal daily dose and supplementation timing of rLH may resolve the debate regarding its efficacy in increasing the number of pregnancies and neonatal survival rates.

## Introduction

In Italy, as well as in the majority of developed countries, the number of females bearing children during the third and fourth decades of life is increasing, as it is common to postpone marriage and pregnancy due to career priorities and advancing education, increased access to contraception and artificial abortion, and financial concerns (1). Therefore, numerous couples, suffering from age-related infertility due to a diminished ovarian reserve (OR), turn to assisted reproductive technologies.

The age related effect on female fertility has been demon strated in several studies concerning *in vitro* fertilization (IVF) treatment in infertile couples, and reports suggest that the success rate decreases in females aged >35 years (2).

When reduced OR is identified, particularly in patients of advanced age, the probability of an insufficient ovarian response, which leads to cycle cancellation, or oocyte retrieval is high. This condition usually occurs in 9–24% of females undergoing IVF treatment, and a significant proportion of these occur in patients, who are considered 'estimated poor responders' (EPRs) (2–4).

In a previous survey of EPR patients from 196 centres in 45 countries, a gonadotropin-releasing hormone (GnRH)-antagonist (ant) regimen was used in 53% of IVF cycles, a short GnRH agonist regimen was used in 20%, a GnRH agonist micro-dose flare regimen was used in 15% and a long GnRH agonist regimen was used in 9% (5,6).

The most common disadvantage in the GnRH-ant method appeared to be the rapid and significant suppression of pituitary function following the administration of GnRH-ant. Although the use of GnRH-ant is limited in the last days of gonadotropin ovarian stimulation, particularly using a flexible scheme, a decline in serum luteinizing hormone (LH) and estradiol (E2) negatively affects the number and quality of oocytes retrieved and, subsequently, the quality of the embryo, resulting in a poor IVF success rate (5).

Physiologically, the activity of LH is relatively low during the menstrual period and progressively increases throughout the mid- to late-follicular phase. During this phase, LH induces granulosa cell growth and differentiation by promoting local peptide synthesis and release, induces the production of epidermal growth factor (EGF) in the thecal interstitial cells and indirectly promotes E2 release by thse granulosa cells (7).

Shimada *et al* (7) demonstrated that the LH peak, inducing the prostaglandin E2 and progesterone dependent pathways in the granulosa cells, mediates critical events during the ovulation process, including reprogramming of the gene expression of the granulosa and cumulus cells during the ovulatory cascade, which affects cumulus expansion and oocyte maturation.

Despite a previous study, performed in unselected patients, failing to detect advantages and often reporting contradictory results of recombinant LH (rLH) supplementation during treatment using recombinant follicle stimulating hormone (rFSH), there is now evidence that rLH supplementation improves the qualitative and quantitative ovarian response, embryo quality and the fertility rate in a selected cohort of patients (8).

A meta-analysis by Alviggi *et al* (8) identified this cohort in patients at risk for poor responsiveness, exhibiting hypo-response to rFSH alone with advanced reproductive age, treated with GnRH-ant.

At present, to the best of our knowledge, no investigations have been performed in this cohort of patients to identify the optimal daily dose of rLH and optimal timing of supplementation during ovarian stimulation.

The aim of the present study was to establish the optimal timing, between the beginning of FSH administration and the beginning of GnRH-ant administration, and the optimal dose (75 IU, vs. 150 IU) of rLH administration in EPR infertile females undergoing IVF cycle using GnRH-ant, in order to achieve the greatest number of retrieved oocytes, optimal oocyte maturation degree and fertilization rate, optimal embryo quality, optimal endometrial thickness at embryo-transfer and the highest pregnancy rate.

## Patients and methods

### Patient information

A pilot cross-matched study was performed on female patients undergoing two fresh, non-donor IVF cycles for primary infertility, with rLH supplementation during ovarian stimulation. The investigation was performed between July 2012 and July 2013 at the Assisted Reproductive Unit of the Gynecological and Obstetrics Clinic, Department of Women's and Children's Health of Padua University (Padua, Italy).

All enrolled patients were informed of the aim of the investigation and they consented to the use of their data, according to the Italian Law for Privacy 675/96 (http://www.garanteprivacy.it/web/guest/home/docweb/-/docweb-display/export/1311248). All patients agreed to the pilot investigation and provided written informed consent, which was obtained at enrolment.

Following consultation of the Local Ethical Committee, the present study was defined exempt from an Institutional Review Board, as rLH supplementation is routinely performed in the Assisted Reproductive Unit of Gynecologic and Obstetrics Clinic, Department of Women's and Children's Health of Padua University, according to the internal treatment instructions, and the pilot nature of the investigation.

The predominant focus of the EPR cohort of patients was their ovarian biological age, rather than their chronological age, as suggested by the Bologna Criteria (2,3).

### Inclusion/Exclusion criteria

Patients were excluded if they had a history of smoking in the previous 6 months, deep endometriosis with an elevated CA125 serum value (9), a previous ART cycle in the last three months, a body mass index (BMI) >30, abnormalities of karyotype, mutations of the cystic fibrosis gene, acquired or inherited thrombophilia or immunological disorders, previous chemotherapy and/or radiotherapy treatment for cancer, untreated uterine diseases, including endometrial polyps, submucous myomas, intrauterine synechiae and/or uterine septum (10,11) or severe qualitative and quantitative alterations in semen (according to World Health Organization guidelines) (12). Patients were also excluded if they had a basal serum LH level >1.2 IU prior to the beginning of treatment and those who received low-dose aspirin during treatment (13). In order to avoid a possible bias in evaluating the pregnancy rate, patients with a personal history of diabetes and thyroid disorders were also excluded (14,15).

### Clinical intervention

All patients underwent GnRH-ant flexible short-regimen stimulation, according to the methods of the Assisted Reproductive Unit of Gynecologic and Obstetrics Clinic, Department of Women's and Children's Health of Padua University. All stimulation cycles were performed using rFSH (*Gonal F^®^*; *Merck-Serono*, *Geneva*, *Switzerland*) at 300 IU/day, beginning from the second day of the menstrual cycle and continuing for 5 days. The subsequent dose adjustments were determined by the clinicians during the cycles, according to the biochemical and ultrasound features of the ovarian response, using transvaginal sonography (TVS; Voluson e6 compact; GE Healthcare, GE Medical Systems, Ltd., Hertfordshire, UK).

On the sixth day of stimulation, all the patients were monitored by hormonal serum sampling (17β estradiol, progesterone and LH) and pelvic ultrasound evaluation. The GnRH-ant (Cetrotide^®^; Industria Farmaceutica Serono, Rome, Italy) at 0.25 mg was administered daily, starting from the TVS detection of at least one follicle measuring >14 mm in diameter, and was continued until human chorionic gonadotropin (hCG) administration.

When an adequate number of follicles (at least three follicles >18 mm in diameter) were observed, 250 *μ*g recombinant hCG (Ovitrelle^®^; Merck-Serono) was administered to induce ovulation.

Oocyte retrieval was performed in theatre 35 h after hCG administration. The oocytes were fertilized using an intracytoplasmic sperm injection technique. On day 3 following retrieval, the obtained embryos were transferred, ensuring to transfer three embryos, when obtained.

Pregnancy was confirmed by an increased concentration of β-hCG 2 weeks after embryo transfer (ET), and TVS detection of an intrauterine gestational sac 3–4 weeks after ET. Ongoing pregnancy was defined by the detection of an embryonic heart beat at the TVS assessment 5–6 weeks following the ET.

As luteal support, vaginal progesterone 200 mg (Progeffik^®^, Effik Italia, Milan, Italy) was administered three times daily until day 14 after retrieval, terminating the treat ment in the case of a negative β-hCG serum test (16).

### Study protocol

At the first cycle, all eligible patients were semi-randomized into group A and group B, by progressively and alternatively assigning patients to a group on recruitment, in order to examine a different daily dose of rLH supplementation.

The patients in group A received 75 IU rLH (Luveris^®^; Merck-Serono). This group was subsequently randomized 1:1 into two subgroups, based on the timing of rLH supplementation: Subgroup A1 received the first rLH dose (75 IU) in concomitance with GnRH-ant (variable day of the cycle) and subgroup A2 received the first rLH dose (75 IU) in concomitance with rFSH administration (second day of the cycle).

The patients in group B received 150 IU rLH. As with group A, group B was also randomized 1:1 into two subgroups: Subgroup B1 received the first rLH dose in concomitance with GnRH-ant and subgroup B2 which received the first rLH dose in concomitance with rFSH administration.

At the second cycle, performed 3 months later, patients who had not become pregnant in the first cycle were reassigned to the alternate group, with patients originally in group A reassigned to group B and vice versa, and were subsequently randomized into subgroup A1/A2 or subgroup B1/B2, as in the first treatment cycle.

### Data collection

For all patients, the following data were collected: Age, body mass index (BMI), total dose of rFSH and rLH administration, days of rLH supplementation, serum levels of 17β E2 and progesterone at hCG administration, number of follicles >10 mm at GnRH-ant administration, number of total follicles and number of follicles measuring >16 mm at hCG administration, endometrial thickness at retrieval, total number of oocytes retrieved, numbers of oocytes at the mature (MII); immature (MI) and germinal vesicle (GV) stages, number of oocytes fertilized, number of embryos obtained, quality of embryos obtained and pregnancy rate. According to Son *et al* (17) and Khoudja *et al* (18), embryos were classified as good, intermediate or poor quality on the basis of the blastomere number, difference in size and degree of fragmentation.

### Endpoints

The primary aim of the present study was to assess differences in all subgroups in follicular growth and the number and quality of oocytes retrieved/embryos obtained and their association with the timing and dose of rLH supplementation.

The secondary aim was to compare patients who had received a low total dose of rLH (<500 IU; termed cohort 1), an intermediate total dose (500-1200 IU; cohort 2) and a high total dose (>1,200 IU; cohort 3) in terms of follicular growth and the number and quality of oocytes retrieved/embryos obtained.

In addition, the effect of the two treatment procedures and the timing of rLH administration were evaluated in terms of endometrial thickness at retrieval and the pregnancy rate.

### Statistical analysis

Statistical analysis was performed using SPSS software version 19 (SPSS, Inc., Chicago, IL, USA) for Windows using parametric and nonparametric tests, where appropriate. The Kolmogorov-Smirnov test was performed to assess the normality of the distribution. Continuous data were assessed using Student's t test for two independent groups (general features). Analysis of variance and Bonferroni's post-hoc test were used to compared data from three or more subgroups. Categorical variables were assessed using a χ^2^ test or Fisher's exact test, where appropriate. The results obtained from the data collection are expressed in absolute numbers and percentages for discrete variables and as the mean ± standard deviation for continuous variables. P<0.05 was considered to indicate a statistically significant difference.

## Results

In the interval duration for the present study, a total of 40 patients were classified as eligible for involvement. Among these, 20 patients were assigned to group A, with 10 patients in subgroup A1 and 10 in subgroup A2, and 20 patients were assigned to group B, with 10 patients in subgroup B1 and 10 in subgroup B2. The two groups and the four subgroups were matched in terms of age, BMI, basal FSH, anti-mullerian hormone, 17β estradiol and antral follicle count (Table I).

In the first and second IVF cycles, no differences were identified between the subgroups in the duration of stimulation or the total dose of rFSH (Table II).

In the first cycle, statistically significant differences were identified between subgroups A1 and B, compared with A2 and B2 regarding the number of follicles measuring >10 mm at GnRH-ant administration (P<0.001) and the number of follicles measuring >16 mm at hCG administration (P<0.001). However, no differences were observed between the subgroups in the total number of follicles at hCG administration. Notably, at hCG administration, subgroup B1 exhibited the highest mean E2 serum value (P<0.001), while subgroup B2 exhibited the highest mean progesterone serum value (P<0.001). On the day of retrieval, subgroup B2 exhibited increased endometrial thickness, compared with subgroup A1 (P<0.001). A similar trend was observed in the second IVF cycle (Table III).

Comparison among the subgroups in the quantitative/qualitative ovarian response revealed a greater number of retrieved oocytes and MII oocytes that patients in the subgroup B1, compared with those in the other subgroups, with a consequently lower number of MI/GV oocytes (P<0.001). In the remaining subgroups, a higher number of total oocytes and MII oocytes were identified in subgroup A1, compared with subgroups A2 and B2 (P<0.01).

Similar statistical difference, to those described above were found between the subgroups in the number of embryos obtained, with the highest number of embryos obtained in subgroup B1 and the lowest number obtained in subgroup A2. This trend was also observed in the second IVF cycle (Table IV).

Concerning the quality of the 165 embryos obtained from the two treatment groups, 88 grade 1 embryos (53.3%), 65 grade 2 embryos (39.3%) and 12 grade 3 embryos (7.4%) were identified. For each single treatment, 1.16±1.0 grade 1 embryos, 0.88±0.7 grade 2 embryos and 0.16±0.4 grade 3 embryos (Table Va) were detected.

Statistically significant differences were found between the subgroups in embryo grading for grade 1 (P<0.001) and grade 2 (P<0.05), but not for grade 3 (Table Va).

Following the first treatment cycle, only five patients, all of which were in subgroup B1, produced more than three embryos. This included four patients producing four embryos and one patient producing five embryos. Following the second treatment cycle, seven patients, all in subgroup B1, produced more than three embryos; five producing four embryos and two producing five embryos.

In terms of pregnancy rates, five (13.5%) patients became pregnant following the first treatment cycle. This limited number of patients did not enable the detection of statistical differences between the subgroups, although three of the five pregnancies (60%) were in subgroup B1, while the remaining two pregnancies were in subgroup A1 (20%) and subgroup B2 (20%), respectively (Table Vb).

Regarding the pregnancy rate of the 35 patients who underwent the second IVF cycle, four patients (12.5%) became pregnancy. In this case, two of the four pregnancies (50%) were in subgroup B1, while the remaining two preg nancies were in subgroup A1 (25%) and subgroup B2 (25%), respectively (Table Vb).

In the stratified data of the total rLH dose administered in all treatments, no significant differences were observed between cohorts 1, 2 or 3, in terms of the total number of follicles at hCG administration (6.1±1.6, vs. 6.3±1.7, vs. 5.9±2.0, respectively). Notably, subgroup B1 exhibited the optimal results (7.0±1.52) and the results in subgroups B1 and A1 were better than those in subgroups B2 and A2 in all of the cohorts (Fig. 1).

Similar to the results obtained from the total number of follicles at hCG administration, no significant differences were observed in the stratified data of the number of follicles with a diameter >16 mm at hCG administration, the total number of oocytes retrieved, and the number of MII oocytes exhibited between the cohorts. The optimal results were identified in subgroup B1, and subgroups B1 and A1 exhibited better results than subgroups B2 and A2 in all cohorts (Figs. 2–4).

In contrast to the aforementioned findings, the stratified data of the endometrial thickness at retrieval revealed a statistically significant difference between the three cohorts, with the optimum results obtained in cohort 3 and the poorest results obtained in cohort 1 (P<0.001). Therefore, endometrial thickness, in contrast to the ovarian response, appeared to exhibit a greater rLH dose-dependent effect than a time-dependent effect (Fig. 5).

## Discussion

During IVF treatment, controlled ovarian hyperstimulation is largely performed using rFSH in combination with a GnRH analogue for the prevention of premature LH surges. However, the use of GnRH analogues deprive the growing follicles of LH, which can affect the qualitative and quantitative ovarian response, as described in the 'two cell two gonadotropin' theory', LH is required to provide the granulosa cells with androgen precursors for estradiol biosynthesis by FSH, for the resumption of meiosis and for progesterone production following ovulation to sustain the endometrium (19).

Clinical data from the ovarian stimulation suggested that the majority of the normo-gonadotrophic females achieved adequate multi-follicular growth by the administration of rFSH alone since, following pituitary downregulation, the residual quantity of LH in this cohort appeared capable of sustaining the local follicular activities required for growth and dominance (8).

By contrast, in the EPR patients treated using GnRH-ant in the present study, rLH supplementation appeared to increase the ovarian response.

To the best of our knowledge, there are limited reports regarding rLH supplementation in short GnRH-an-treated EPR patients. In addition, the optimal timing of rLH supplementation and its optimal daily dose remains to be elucidated.

De Placido *et al* (20) found that, in a cohort of EPR patients treated using the short GnRH-ant method, rLH supplementation of 150 IU/day at GnRH-ant administration resulted in a higher number of MII oocytes, compared with the patients treated using the short GnRH-agonist with the same total dose of rLH supplementation.

Bosh *et al* (21) found that, in a cohort of patients with normal ovulation cycles treated with GnRH-ant, rLH supplementation (75 IU) significantly increased the implantation rate, but not the pregnancy rate in females aged >35 years.

By contrast, in a study by König *et al* (22), rLH adminis tration demonstrated no improvements in ovarian response or implantation/pregnancy rate in patients aged >35 years treated with GnRH-ant.

Although all the patients received rFSH and rLH in the present study, initial analysis of the data revealed differences in ovarian response, and the quality and number of oocytes and embryos depending on the timing and daily dose of administration. In particular, there was a significant improvement in the two subgroups that received rLH supplementation at GnRH-ant administration, compared with the subgroups, which received rLH on the first day of stimulation.

LH supplementation at GnRH-ant administration compensates for the severe drop in levels of endogenous LH due to administration of the antagonist itself. In addition, it produces a gonadotrophic environment more similar to the physiological environment. During IVF treatment, compared with the physiological cycle, an LH surge is not necessary to select the dominant follicle, however, its activity on the molecular cascade of the granulosa cells persists and remains a fundamental step in achieving a suitable ovarian response and to induce the meiotic division of oocytes (23,24).

However, in GnRH-ant treatment, the co-administration of FSH and LH from the second day of the menstrual cycle produces an excess of LH, derived from endogenous and exogenous components. The concept of an 'LH ceiling' has been widely discussed, which refers to the maximum LH serum level, above which the follicle is no longer stimulated. It is important to underline that each follicle has a different ceiling 'ceiling' level, which depends on its developmental stage. For this reason, the same LH value may be below the ceiling dose for certain follicles, promoting their growth, and above the ceiling dose for other smaller follicles, causing atresia (25).

This concept explains why, when LH was administered in the early stages of follicular growth in the present study, a lower number of follicles measuring >10 mm at GnRH ant administration, a lower number of follicles measuring >16 mm at ovulation induction, and a lower number of retrieved oocytes were observed, compared with administration at a later stage..

The data of the present study revealed no significant differ ences between the subgroups in terms of the total number of follicles at ovulation induction.

These findings can be explained by evidence suggesting that the number of growing follicles recruited depends on the quantity of available follicles (ovarian reserve) and by the growth stimulus provided by FSH alone. However, the degree of maturity of the retrieved oocytes was different in these follicles, and this may be a direct effect of the timing and dose of rLH supplementation.

During controlled ovarian stimulation, the concept of 'FSH windows' is exceeded due to the continuous high dose of rFSH administration in association with the absence of negative pituitary feedback. This enables the recruitment and support of all 'responder' follicles until the pre ovulatory phase. Therefore, the substrate of FSH action depends only on the number of primordial and primary follicles available in the ovarian cortex at the beginning of the cycle (26).

Concerning oocyte quality, Ruvolo *et al* (27) found a lower rate of cumulus cell apoptosis in patients treated with rFSH and rLH. Similarly, Barberi *et al* (28) demonstrated that patients undergoing stimulation with rFSH supplemented with rLH in the late follicular phase achieved a higher concentration of RNA expression in the cumulus cells and higher intra-follicular levels of numerous growth factors.

The two above-mentioned authors hypothesized that rLH supplementation results in an improved follicular environment, enabling a comparable degree of oocyte growth and maturation to that usually detected in young normal responders. The data of the present study were in agreement with these findings, suggesting that a adequate oocyte quality was achieved when rLH was administered in the mid-follicular phase and positively affected the number and quality of embryos obtained. Concerning hormonal patterns, the E2 serum level detected in subgroup B1 confirmed that the mid-follicular phase was optimal for the timing of rLH supplementation to obtain a good quantitative and qualitative ovarian response. By contrast, the higher level of progesterone, observed in patients who received a high dose of rLH (subgroup B2) confirmed the positive rLH dose-dependent effect on endometrial thickening. It is well-established that the endometrial implantation window is crucial to achieve optimal implantation and pregnancy rates, however, the association between the endometrial thickness and the implantation window remains to be elucidated. Routinely, clinicians attempt to avoid areas of the endometrium that are too thin or thick at retrieval, in order to reduce the risk of low implantation rate due to the event of embryo-transfer prior to or following the implantation windows (16). Kolibianakis *et al* (29) performed several investigations regarding the role of serum levels of LH and the implantation rate, reporting that high LH levels in the early follicular phase, which increases the production of estrogen by androgens, anticipates the implantation window and increases the risk of 'post-mature' endometrium at ovulation, reducing the implantation rate. It has been demonstrated that a discrepancy of >3 days between ovulation and the implantation window markedly reduces the implantation rate and, consequently, the chances of becoming pregnant (30,31). However, despite confirming that a high dose of rLH supplementation increased the endometrial thickness at retrieval, the results of the present study cannot determine whether this is a clinical advantage, as the overall number of pregnancies achieved were insufficient and the patients who received a higher dose of rLH were often administered the supplement at the beginning of the stimulation.

The strengths of the present study included the selection of the patient cohort, which appeared to be appropriate for rLH supplementation during the IVF cycle, the strict inclusion criteria and the homogeneity between the groups and subgroups for general features, minimization of possible selection bias and the use of the same stimulatory methods for all treatments, with the exceptions of inevitable dose-adjustments during stimulation. The present study is the first investigation, to the best of our knowledge, with the aim of detecting the optimal dose and timing of rLH supplementation in EPR patients, however, it was not without limitations. The limitations included the limited sample size, and the low ovarian response and pregnancy rates due to the features of the patients and the lack of data regarding the possible differences in intra-follicular growth factors. These factors not enable the true estimation of the differences between the groups and subgroups in terms of pregnancy rate, ongoing pregnancy and the neonatal survival rate.

According to the available data, EPRs undergoing IVF cycles using GnRH-ant may benefit from rLH supplementation. The optimal timing to administer rLH appeared to be the mid-follicular phase, which, in a large proportion of cases, corresponded with GnRH-ant administration.

The optimal quantitative and qualitative ovarian response, and the embryo quality were achieved by using rLH (150 IU/day) independently from the total administered dose.

Regarding the effects on the endometrium of rLH supplementation, the total dose had a greater effect than the timing of administration in improving endometrial thickness. However, its impact on the improvement of pregnancy rate remains to be elucidated.

In addition a larger range of treatments may be required in this cohort of patients to fully understand the role of rLH supplementation in increasing the chances of becoming preg nant in patients with EPR.

## Figures and Tables

**Figure 1:** Total number of follicles at hCG administration. Stratification data between the subgroups and cohorts (recombinant luteinizing hormone supplementation: daily dose, vs. timing, vs. total dose). hcg, human chorionic gonadotropin.

**Figure 2:** Number of follicles measuring >16 mm at hCG administration. Stratified data between the subgroups and cohorts (recombinant luteinizing hormone supplementation: daily dose, vs. timing, vs. total dose). hcg, human chorionic gonadotropin.

**Figure 3:** Total number of oocytes retrieved. Stratified data between the subgroups and cohorts (recombinant luteinizing hormone supplementation: daily dose, vs. timing, vs. total dose).

**Figure 4:** Number of MII oocytes: stratification data between the subgroups and cohorts (recombinant luteinizing hormone supplementation: daily dose, vs. timing, vs. total dose).

**Figure 5:** Endometrial thickness at oocyte retrieval: stratification data between the subgroups and cohorts (recombinant luteinizing hormone supplementation: daily dose, vs. timing, vs. total dose).

**Table I:** General features of participants in the study: Comparison between groups and subgroups.

Variable	No. patients (n)	Mean ± SD	Range	Subgroup (n)	Mean ± SD
1^st^ IVF cycle					
Age	40	40.3±1.48	37-42	A1 (10)	40.4±1.58
				A2 (10)	40.5±1.58
				B1 (10)	40.2±1.39
				B2 (10)	40.1±1.59
Body mass index	40	23.1±1.60	20-25	A1 (10)	23.0±1.89
				A2 (10)	23.2±1.62
				B1 (10)	23.4±1.43
				B2 (10)	22.9±1.66
b-FSH (IU/l)	40	12.7±2.30	8.1-16.4	A1 (10)	12.7±2.48
				A2 (10)	13.6±2.13
				B1 (10)	12.2±1.81
				B2 (10)	12.3±2.75
b-AMH (*μ*g/l)	40	0.5±0.28	0.1-0.9	A1 (10)	0.5±0.29
				A2 (10)	0.5±0.29
				B1 (10)	0.6±0.27
				B2 (10)	0.5±0.28
b-17β estradiol (nmol/l)	40	0.2±0.06	0.29-0.19	A1 (10)	0.2±0.06
				A2 (10)	0.2±0.06
				B1 (10)	0.2±0.05
				B2 (10)	0.2±0.05
Antral follicle count	40	5.0±1.86	2-9	A1 (10)	4.8±1.81
				A2 (10)	4.3±1.77
				B1 (10)	5.9±1.85
				B2 (10)	5.2±1.93
2^nd^ IVF cycle					
Age	35	40.3±1.55	37-42	A1 (8)	39.6±1.59
				A2 (8)	40.7±1.39
				B1 (10)	40.2±1.68
				B2 (9)	40.6±1.50
Body mass index	35	23.2±1.58	20-25	A1 (8)	23.7±1.28
				A2 (8)	23.0±1.51
				B1 (10)	22.7±1.63
				B2 (9)	23.6±1.80
b-FSH (IU/l)	35	12.5±2.19	9.2-16.0	A1 (8)	12.8±2.32
				A2 (8)	13.3±2.05
				B1 (10)	12.3±2.18
				B2 (9)	11.8±2.31
b-AMH (*μ*g/l)	35	0.4±0.28	0.1-0.9	A1 (8)	0.5±0.28
				A2 (8)	0.3±0.31
				B1 (10)	0.5±0.22
				B2 (9)	0.4±0.29
b-17β estradiol (nmol/l)	35	0.2±0.06	0.11-0.29	A1 (8)	0.2±0.05
				A2 (8)	0.2±0.06
				B1 (10)	0.2±0.06
				B2 (9)	0.2±0.07
Antral follicle count	35	4.5±1.85	2-9	A1 (8)	5.1±1.72
				A2 (8)	3.6±1.50
				B1 (10)	4.9±2.08
				B2 (9)	4.5±1.94

SD, standard deviation; b-, basal; FSH, follicle stimulating hormone; AMH, anti-mullerian hormone; IVF, *in vitro* fertilisation.

**Table II:** Comparison of the duration of ovarian stimulation and total dose of rFSH between groups and subgroups.

Variable	No. patients (n)	Mean ± SD	Range	Subgroup (n)	Mean ± SD
1^st^ IVF cycle					
Duration of rFSH administration (days)	40	11.4±1.25	9-13	A1 (10)	11.4±1.26
				A2 (10)	11.2±1.39
				B1 (10)	11.5±1.43
				B2 (10)	11.4±1.07
Total dose of rFSH administered (IU)	40	3,875.0±702.85	2,475-5,200	A1 (10)	3,922.5±649.62
				A2 (10)	3,830.0±750.53
				B1 (10)	3,895.0±858.03
				B2 (10)	3,852.5±644.96
2^nd^ IVF cycle					
Duration of rFSH administration (days)	35	10.6±1.19	9-13	A1 (8)	10.5±1.19
				A2 (8)	10.5±1.19
				B1 (10)	10.9±1.29
				B2 (9)	10.5±1.24
Total dose of rFSH administered (IU)	35	3,652.1±538.80	2,700–4,875	A1 (8)	3,650.0±662.92
				A2 (8)	3,681.2±514.04
				B1 (10)	3,700.0±560.88
				B2 (9)	3,575.0±503.74

No significant differences were identified. rFSH, recombinant follicle stimulating hormone; IVF, *in vitro* fertilisation; SD, standard deviation.

**Table III:** Comparison of transvaginal sonography and hormonal response, and endometrium between groups and subgroups.

Variable	No. patients (n)	Mean ± SD	Range	Subgroup (n)	Mean ± SD	P-value
1^st^ IVF cycle						
Follicles >10 mm at GnRH- ant administration (n)	40	3.3±1.42	1-6	A1 (10)	4.1±1.29^a^	<0.001
				A2 (10)	2.1±0.74^b^	
				B1 (10)	4.5±0.85^c^	
				B2 (10)	2.5±1.08^d^	
Total follicles at hCG administration (n)	40	5.9±1.96	3-9	A1 (10)	6.0±2.00	n.s.
				A2 (10)	5.2±1.75	
				B1 (10)	7.2±1.75	
				B2 (10)	5.1±1.85	
Follicles >16 mm at hCG administration (n)	40	2.9±1.37	1-6	A1 (10)	3.2±1.13^e^	<0.001
				A2 (10)	2.2±0.79^f^	
				B1 (10)	4.5±1.08^g^	
				B2 (10)	2.0±0.81^h^	
Serum value of 17β estradiol at hCG day (nmol/l)	40	5.1±1.78	2.45-9.05	A1 (10)	4.3±1.11^i^	<0.001
				A2 (10)	3.9±0.69^j^	
				B1 (10)	7.7±0.94^k^	
				B2 (10)	4.3±0.81^l^	
Serum value of progesterone at hCG day (nmol/l)	40	3.0±0.75	1.59-4.76	A1 (10)	2.2±0.32^m^	<0.001
				A2 (10)	3.2±0.60^n^	
				B1 (10)	3.0±0.50^o^	
				B2 (10)	3.6±0.64^p^	
Endometrial thickness at retrieval (mm)	40	11.8±1.49	11.3-12.2	A1 (10)	10.2±0.41^q^	<0.001
				A2 (10)	11.5±0.74^r^	
				B1 (10)	11.4±0.93^s^	
				B2 (10)	13.8±0.68^t^	
2^nd^ IVF cycle						
Follicles >10 mm at GnRH- ant administration (n)	35	3.4±1.40	1-6	A1 (8)	4.0±1.60^a^	<0.01
				A2 (8)	2.4±1.06^b^	
				B1 (10)	4.4±0.85^c^	
				B2 (9)	2.9±0.78^d^	
Total follicles at hCG administration (n)	35	6.4±1.54	3-9	A1 (8)	6.5±1.51	n.s.
				A2 (8)	6.2±1.49	
				B1 (10)	6.8±1.32	
				B2 (9)	6.1±1.96	
Follicles >16 mm at hCG administration (n)	35	3.2±1.35	1-6	A1 (8)	3.5±1.07^e^	<0.001
				A2 (8)	2.5±0.75^f^	
				B1 (10)	4.6±1.07^g^	
				B2 (9)	2.1±0.78^h^	
Serum value of 17β estradiol at hCG day (nmol/l)	35	4.9±1.55	1.60-8.10	A1 (8)	5.0±1.37^i^	<0.01
				A2 (8)	4.0±1.15^j^	
				B1 (10)	6.1±1.20^k^	
				B2 (9)	4.2±1.57^l^	
Serum value of progesterone at hCG day (nmol/l)	35	3.1±0.76	1.52-4.35	A1 (8)	2.3±0.48^m^	<0.001
				A2 (8)	3.1±0.56^n^	
				B1 (10)	2.9±0.57^o^	
				B2 (9)	4.0±0.24^p^	
Endometrial thickness at retrieval (mm)	35	11.9±1.58	11.3-12.5	A1 (8)	10.4±1.01^q^	<0.001
				A2 (8)	11.2±1.00^r^	
				B1 (10)	12.1±1.10^s^	
				B2 (9)	13.7±1.09^t^	

1st IVF cycle Bonferroni post-hoc test: P<0.01, a vs, b,d; P<0.001, b vs, c; P<0.01, c vs, d; P<0.001, e vs, g,h; P<0.05, e vs, f; P<0.001, k vs, i,j,l; P<0.001, m vs, n,p; P<0.01, m vs, o; P<0.01, q vs r,s; P<0.001, q vs, t; P<0.001, r vs, t; P<0.001, s vs, t. 2nd IVF cycle Bonferroni post-hoc test: P<0.001, b vs, c; P=0.054, a vs, b,c,d; P<0.001, e vs g,h; P<0.05, f vs, h; P<0.05, k vs, j,l; P<0.001, p vs, m,o; P<0.01, p vs, n; P<0.05, n vs, m; P<0.001, t vs, q,r; P<0.05, t vs, s; P<0.05, q vs, s. IVF, *in vitro* fertilization; SD, standard deviation; n.s., not significant.

**Table IV:** Data regarding quantitative/qualitative ovarian response and embryos obtained following ICSI technique: Comparison between groups and subgroups.

Variable	No. patients (n)	Mean ± SD	Range	Subgroups (n)	Mean ± SD	P-value
1^st^ IVF cycle						
Total oocytes retrieved (n)	40	3.9±1.46	2-7	A1 (10)	4.2±1.13^a^	<0.001
				A2 (10)	2.6±0.52^b^	
				B1 (10)	5.7±0.95^c^	
				B2 (10)	3.1±0.74^d^	
MII oocytes (n)	40	2.9±1.48	0-6	A1 (10)	3.1±0.74^e^	<0.001
				A2 (10)	1.6±0.70^f^	
				B1 (10)	4.9±0.74^g^	
				B2 (10)	2.0±0.82^h^	
MI/GV oocytes (n)	40	1.0±0.68	0 -2	A1 (10)	1.1±0.74	n.s.
				A2 (10)	1.0±0.67	
				B1 (10)	0.8±0.63	
				B2 (10)	1.1±0.74	
Total embryos obtainedafter ICSI (n)	40	2.0±1.19	1.67-2.43	A1 (10)	2.1±0.74^i^	<0.001
				A2 (10)	1.1±0.74^j^	
				B1 (10)	3.6±0.70^k^	
				B2 (10)	1.4±0.70^l^	
2^nd^ IVF cycle						
Total oocytes retrieved (n)	35	3.9±1.50	1-7	A1 (8)	4.1±1.24^a^	<0.001
				A2 (8)	2.8±0.99^b^	
				B1 (10)	5.4±1.07^c^	
				B2 (9)	3.2±1.30^d^	
MII oocytes (n)	35	2.8±1.57	0-6	A1 (8)	3.0±0.92^e^	<0.001
				A2 (8)	1.5±0.75^f^	
				B1 (10)	4.7±0.95^g^	
				B2 (9)	1.9±1.05^h^	
MI/GV oocytes (n)	35	1.1±0.63	0 -2	A1 (8)	1.1±0.64	n.s.
				A2 (8)	1.4±0.52	
				B1 (10)	0.7±0.67	
				B2 (9)	1.3±0.50	
Total embryos obtainedafter ICSI (n)	35	2.4±1.28	1.93-2.81	A1 (8)	2.4±0.74^i^	<0.001
				A2 (8)	1.5±0.75^j^	
				B1 (10)	3.8±0.92^k^	
				B2 (9)	1.6±1.01^l^	

1st IVF Cycle Bonferroni post-hoc test: P<0.001, c vs, b,d; P<0.01, c vs, a; P<0.01, a vs, b; P<0.05, a vs, d; P<0.001, g vs, e,f,h; P<0.001, e vs, f; P<0.05, e vs, h; P<0.001, k vs, i,j,l; P<0.05, i vs, j. 2^nd^ IVF cycle Bonferroni post-hoc test: P<0.001, c vs, b; P<0.01, c vs, d; P<0.001, g vs, f,h; P<0.01 g vs,e; P<0.05, e vs, f; P<0.001, k vs, j,l; P<0.05, k vs, i. IVF, *in vitro* fertilization; SD, standard deviation; ICSI, intracytoplasmic sperm injection; MII, mature; MI, immature; GV, germinal vesicle; n.s., not significant.

**Table V:** Embryos, pregnancy and their stratification according to groups and sub-groups of treatment.

A, Embryo quality and stratification according to treatment groups and subgroups (considering 1st and 2nd IVF cycles)							
Patient	Grade 1 embryos		Grade 2 embryos		Grade 3 embryos		Total number
	Number	%	Number	%	Number	%	
Subgroup							
A1	22^a^	55.0	15	37.5	3	7.5	40
A2	9^b^	39.1	10^e^	43.5	4	17.4	23
B1	48^c^	64.9	24^f^	32.4	2	2.7	74
B2	9^d^	32.1	16	57.1	3	10.8	28
Total embryos (n)	88	53.3	65	39.3	12	7.4	165

B, Pregnancies and stratification according to treatment groups and subgroups					
Patient	Not pregnant		Pregnant		Total number
	Number	%	Number	%	
1^st^ IVF cycle					
Subgroup					
A1	9	90.0	1	10.0	10
A2	8	100.0	0	0.0	8
B1	7	70.0	3	30.0	10
B2	8	88.9	1	11.1	9
Total for grade	32	86.5	5^a^	13.5	37
2^nd^ IVF cycle					
Subgroup					
A1	7	87.5	1	12.5	8
A2	7	100.0	0	0.0	7
B1	8	80.0	2	20.0	10
B2	6	85.7	1	14.3	7
Total for grade	28	87.5	4^a^	12.5	32

Bonferroni post-hoc test: P<0.001 c vs, a,b,d; P<0.001 a vs, d; P<0.05 a vs, b; P<0.05 f vs, e. IVF, *in vitro* fertilization.
